The article "miR-195 Inhibits Proliferation and Enhances Apoptosis of OSCC Cells via Targeting TLR4" was retracted in 2023. Reasons: signs of a paper mill; suspected computer-generated content; unreliable results or conclusions; lack of ethics approval or compliance.

# miR-195 Inhibits Proliferation and Enhances Apoptosis of OSCC Cells via Targeting TLR4

**DOI:** 10.1155/2022/2270777

**Published:** 2022-03-09

**Authors:** Jianguo Wang, Renyou Song, Chunmei Wang, Shuangsheng Zhang, Yanqi Zhang, Yanlong Zhu, Gang Zhao

**Affiliations:** Department of Oral and Maxillofacial Surgery, Jiamusi University Affiliated Stomatological Hospital, Jiamusi, China

## Abstract

The aim of this research was to assess the function of microribonucleic acid (miR)-195 in the apoptosis and proliferation of oral squamous cell carcinoma (OSCC) cells as well as its action mechanism. The downstream target protein of miR-195 was predicted using the biological software. A quantitative polymerase chain reaction (qPCR) was implemented to examine the changes in expressions of miR-195 and its target protein toll-like receptor 4 (TLR4) in OSCC cell lines (TSCCA, Tca8223, Tb3.1, and CAL-27) and normal adult human gingival fibroblasts (HGFs), and the relation between their expressions was assessed. The expressions of phosphorylated proteins in nuclear factor-*κ*B (NF-*κ*B) pathway were determined through western blotting. miR-195 was expressed at a noticeably lower level in four OSCC cells than in HGFs, and the lowest level appeared in CAL-27 cells. Compared with miR-195 control, the miR-195 mimic could obviously raise the expression of miR-195. In CAL-27 cells with high expression of miR-195, the proliferation was inhibited and the apoptosis was evidently enhanced. OSCC cells exhibited evidently reduced protein and mRNA expression of TLR4, and miR-195 expression was inversely associated with TLR4 expression. It was uncovered from the dual-luciferase reporter assay that cells with wild-type TLR4 had prominently weakened luciferase activity relative to cells with mutant-type TLR4, revealing that the direct target of miR-195 is TLR4. The NF-*κ*B pathway was impeded in cells that lowly expressed TLR4. miR-195 blocks the NF-*κ*B pathway via inhibiting the expression of TLR4 in OSCC cells, thereby exerting an antitumor effect.

## 1. Introduction

As a malignancy of the oral cavity, oral squamous cell carcinoma (OSCC) has a high relapse rate in the clinic, and the five-year survival rate in patients is below 50% [1]. In the past three decades, the five-year survival rate of OSCC patients was below 50% owing to the high relapse and death rates in spite of the remarkable efficiency in surgery and chemoradiotherapy for primary tumors in the oral cavity [2, 3]. There is a necessity to comprehend the molecular mechanisms by which OSCC cells proliferate, invade, and metastasize, which are the basis for relapse, so as to efficaciously treat OSCC.

Microribonucleic acids (miRNAs) are formed during mRNA maturation and consist of about 22 bases, which can silence downstream target mRNAs, thereby inhibiting protein expression and affecting tumor biological processes [4–8]. miRNAs such as miR-145, miR-338, and miR-433 have been verified to influence the invasion, proliferation, and apoptosis (biological phenotypes) as well as the pathological process of OSCC cells [9–11]. It is shown in several reports that the expression of miR-195-5p declines in tumors [12–14]. Jia et al. [15] held that miR-195-5p overexpression probably performs its function in inhibiting the onset and progression of tongue squamous cell carcinoma. Nevertheless, the target gene and mechanism of miR-195-5p in OSCC remain elusive.

Toll-like receptor 4 (TLR4), expressed in macrophages, is a pivotal receptor responding to numerous signaling events in polysaccharide detection [16, 17]. TLR4 is also of great importance for the enhancement of innate immunity and production of cytokines after polysaccharide stimulation [18]. As a transcription factor in cells, nuclear factor-*κ*B (NF-*κ*B) is mainly involved in the inflammatory response, and it can promote cell function and gene expression after activation [19]. The activity of NF-*κ*B is strictly controlled by positive and negative regulators. In the inactive state, NF-*κ*B family members exist as dimers, mainly p65/p50 heterodimers, which are isolated in the cytoplasm by I-*κ*B family members. Through such a dynamic mechanism, the genes are regulated via activating transcription factors, such as NF-*κ*B [20]. In addition, TLR-dependent signaling pathways, after being activated, will affect the phosphorylation activity of mitogen-activated protein kinase, and a cascade reaction will occur among these pathways, ultimately activating transcription factor complexes in nuclei.

The aim of the current research was to explore the effects of miR-195 on the apoptosis and proliferation of OSCC cells and to further investigate the potential underlying molecular mechanism.

## 2. Materials and Methods

### 2.1. Cell Lines

The objects of this study included OSCC TSCCA, Tca8223, Tb3.1, and CAL-27 cells, and transfection with exogenous miR-195 sequences raised miR-195 expression levels in CAL-27 cells. The cells undergoing miR-195 mimic transfection were included in the miR-195 mimic group, while those receiving miR-195 control transfection were enrolled in the miR-195 control group.

### 2.2. Cell Transfection In Vitro

miR-195 mimic and miR-195 control were purchased from Keygen Biotech (Nanjing, China) Company. Before transfection, CAL-27 cells were cultured until 60% of them were fused. According to the instructions, a 50 nM virus solution was prepared and transfected into cells using Lipofectamine 3000 transfection reagent (Invitrogen, Carlsbad, CA, USA). A quantitative polymerase chain reaction (qPCR) was implemented to determine the transfection efficiency.

### 2.3. Real-Time Fluorescence qPCR

The TRIzol reagent from Invitrogen (Carlsbad, CA, USA) was utilized for total RNA extraction in a biosafety cabinet on ice, and the RNA was resuspended in DEPC-treated water bought from Beyotime (Shanghai, China). Then, cDNA was synthesized using the kit. Finally, 20 *μ*L of system was prepared using SYBR Green buffer, followed by qPCR amplification. The relative gene expression was calculated, with U6 as a reference. The primer sequences of miR-195 and phosphorylated NF-*κ*B (p-NF-*κ*B) are as follows: miR-195-F: 5′-ACACTCCAGCTGGGTAGCAGCACAGAAAT-3′; miR-195-R: 5′-TGGTGTCGTGGAGTCG-3′. TLR4-F: 5′-GCCGGAAAGTTATTGTGGTGGT-3′; TLR4-R: 5′-ATGGGTTTTAGGCGCAGAGTTT-3′. p-NF-*κ*B-F: 5′-CCAAAGAAGGACACGACAGAATC-3′; p-NF-*κ*B-R: 5′-GGCAGGCTATTGCTCATCACA-3′. U6-F: 5′-CTCGCTTCGGCAGCACA-3'; U6-R: 5′-AACGCTTCACGAATTTGCGT-3′. GAPDH-F: 5′-GAGTCAACGGATTTGGTCGT-3′; GAPDH-R: 5′-GAGTCAACGGATTTGGTCGT-3′.

### 2.4. Western Blotting

The reagents were thawed on ice before the experiment, and the cells were resuspended in phosphate buffered saline (PBS), which was sucked out after centrifugation. Next, a proper volume of cell lysis buffer was added for 30 min of ultrasonication at 13,000 rpm. The supernatant was aspirated, and the protein concentration was detected at 560 nm. Subsequent to SDS-PAGE in a 10–15% Tris-glycine gel, the protein was transferred onto a membrane for 1 h and sealed for 5 min, followed by rinsing in accordance with standard procedures and 15 h of incubation with primary antibodies (Abcam, Cambridge, MA, USA). The next day, the protein receives a 1 h incubation with secondary antibodies at room temperature. Lastly, Amersham ECL™ reagent from Thermo Fisher Scientific (Waltham, MA, USA) was utilize to visualize the membrane.

### 2.5. Cell Proliferation Assay

3-(4,5-dimethylthiazol-2-yl)-2,5-diphenyl tetrazolium bromide (MTT) assay (Sigma-Aldrich, St. Louis, MO, USA) was carried out to examine cell proliferation changes, briefly as follows: the cells were inoculated into a 96-well plate (3000 cells/well) containing 200 *μ*L of medium. After MTS reagent was added for incubation for 2 h, the absorbance of the cells was measured. The assay lasted for 5 d.

### 2.6. Cell Apoptosis Assay

After culture for 48 h, the cells were collected (the number of dead cells <3%) and prepared into cell suspension with trypsin quickly. Then, the cell suspension was transferred into a centrifuge tube, washed with PBS, and transferred into an Eppendorf (EP) tube, followed by staining with AnnexinV-FITC (fluorescein isothiocyanate) and propidium iodide (PI) for 10 min each in the dark. Finally, the proportion of apoptotic cells was detected using flow cytometry (FACSCalibur; BD Biosciences, Detroit, MI, USA).

### 2.7. Determination of Luciferase Activity

The 3′-untranslated region (3′-UTR) of the TLR4 reporter gene was constructed, which contained a specific miR-195-targeted site and a random scrambling sequence inserted into the pGL3 vectors. It was predicted that the sequence was not a target of miR-195. TLR4 3′-UTR mutant-type and wild-type plasmids were cotransfected with miR-195. Finally, the luciferase activity was determined using the dual-luciferase reporter system at 48 h after cotransfection.

### 2.8. Statistical Analysis

The data were expressed as the mean ± standard deviation in three assays. The correlation between miR-195-5p and TLR4 expressions was detected via the Spearman correlation test. The Statistical Product and Service Solutions (SPSS) 21.0 software (IBM, Armonk, NY, USA) was used, and the *t* test was performed for the comparison between the two groups. *P* < 0.05 suggested a statistically significant difference.

## 3. Results

### 3.1. miR-195 Overexpression Repressed OSCC Cells to Proliferate

The QPCR assay results of the changes in miR-195 expression in OSCC cells unveiled that miR-195 was expressed at a notably lower level in OSCC cells than that in normal HGFs (*P* < 0.05), which was the lowest in CAL-27 cells. miR-195 expression in CAL-27 cells could be elevated following transfection with exogenous miR-195 sequences (*P* < 0.001). Besides, the changes in cell proliferation were detected via the MTT assay, and it was found that the upregulation of miR-195 reduced cell proliferation compared with the negative control (*P* < 0.05) (Figure 1).

### 3.2. Upregulation of miR-195 Promoted Apoptosis

The changes in apoptosis of OSCC cells were detected via flow cytometry. The results showed that the proportion of apoptotic cells in the miR-195 mimic group was evidently higher than that in the miR-195 control group (*P* < 0.05) (Figure 2).

### 3.3. miR-195 and TLR4 Expressions Were Negatively Correlated in OSCC Cells

According to the results of qPCR, miR-195 had markedly lower expression in OSCC cells than that in HGF (*P* < 0.01), while the TLR4 mRNA expression showed the opposite trend in OSCC cells (*P* < 0.05). It was found via Spearman correlation analysis that there was a negative correlation between expressions of miR-195 and TLR4 in OSCC cells (*r*^2^ = 0.79) (*P* < 0.001) (Figure 3).

### 3.4. miR-195 Directly Downregulated the Expression of TLR4 Protein in OSCC Cells

The downstream target protein of miR-195 was predicted through bioinformatics, and the results manifested that miR-195 had binding sites with TLR4 3′-UTR. According to the results of the dual-luciferase reporter assay, there was a 50% reduction in the luciferase activity in CAL-27 cells undergoing wild-type TLR4 transfection, but no basic changes were found in cells receiving mutant TLR4 transfection, manifesting that TLR4 is a target of miR-195 (Figure 4).

### 3.5. Upregulation of miR-195 Blocked the NF-*κ*B Pathway

To detect the effect of miR-195 on the activity of the NF-*κ*B pathway in OSCC cells, the changes in p-NF-*κ*B protein and mRNA expression were determined in cells transfected with miR-195 mimic and miR-195 control. The results manifested that the miR-195 mimic group had remarkably lower p-NF-*κ*B protein and mRNA expression than the miR-195 control group (*P* < 0.01) (Figure 5).

## 4. Discussion

miR-195, a member of the miR-15 family, is associated with thyroid carcinoma, hepatocellular carcinoma, etc. [21]. Furthermore, miR-195 displays low expression in tumors and plays an inverse regulatory role. Given this, it is speculated that miR-195 may also exert an antitumor effect in OSCC cells.

The current research demonstrated that miR-195 was expressed at a prominently lower level in OSCC cell lines relative to that in HGFs. For investigating the biological functions of miR-195 in OSCC cells, miR-195 was overexpressed in CAL-27 cells. After upregulation of miR-195, there were changes in the biological behaviors of CAL-27 cells, such as weakened cell proliferation and enhanced apoptosis, which is exactly the desired therapeutic effect on OSCC. In OSCC, miR-195 exerts an antitumor effect, and it suppresses the formation of malignant phenotypes of OSCC cells after overexpression, suggesting that miR-195 possesses great potential in treatment. Moreover, miRNAs can serve as oncogenes or tumor suppressor genes by interacting with specific targets [22]. TLR4 is reported to participate in the onset of periodontitis, and it is a core factor for the inflammatory response in stroke and other head-associated traumas, so TLR4 expression changes probably exert vital effects in OSCC cells. In the meantime, biological software was utilized to predict miR-195 expression-related target genes in the present research, and TLR4 was verified to be a target gene. Therefore, it is speculated that miR-195 regulates tumor progression via targeting TLR4. In the 4 kinds of OSCC cells, TLR4 had markedly increased expression, while miR-195 showed the opposite trend. Then, the correlation between TLR4 and miR-195 expressions was explored via Spearman correlation analysis, and a negative correlation was confirmed between them, with a significant difference. Meanwhile, according to the results of dual-luciferase reporter assay, cells undergoing wild-type TLR4 transfection had evidently weakened luciferase activity probably because miR-195 silenced the protein expression of TLR4 through binding to wild-type TLR4 3′-UTR. In other words, TLR4 is a direct target gene of miR-195.

TLR4 is able to facilitate inflammatory responses as well as TNF-*α* and IL-1*β* production, and it is also implicated in tissue inflammatory responses requiring nuclear transcription factor NF-*κ*B. The activated TLR4/NF-*κ*B pathway leads to inflammatory response and tumor progression [23]. Therefore, reducing the utilization rate of TLR4 ligand and/or inhibiting TLR4 signal transduction in tumor cells is expected to prevent further aggravation of tumor. The present research manifested that miR-195 overexpression enhanced the phosphorylation of NF-*κ*B in CAL-27 cells, probably because elevating miR-195 repressed TLR4 expression, thereby impeding the TLR4/NF-*κ*B signaling pathway. Therefore, targeting the miR-195/TLR4 interaction can be used as a new therapeutic method for OSCC. However, the difference in miR-195 expression in tissues and the effect of miR-195 on tumor formation were not explored in this study, which, therefore, needs to be researched in the future.

## 5. Conclusions

In conclusion, miR-195 blocks the NF-*κ*B pathway via directly inhibiting the expression of TLR4 in OSCC cells, thereby exerting an antitumor effect.

## Figures and Tables

**Figure 1:** Effect of upregulation of miR-195 on OSCC cell proliferation. (a) miR-195 expression in OSCC cells. The expression of miR-195 is obviously lower in TSCCA, Tca8223, Tb3.1, and CAL-27 cells than that in HGF (*P* < 0.05). (b) Expression of miR-195 in CAL-27 cells after transfection with miR-195 mimic. The expression of miR-195 in CAL-27 cells obviously rises after transfection with miR-195 mimic compared with that after transfection with miR-195 control (*P* < 0.01). (c) Effect of miR-195 on CAL-27 cell proliferation. The absorbance at 490 nm obviously declines in the miR-195 mimic group compared with that in the miR-195 control group (*P* < 0.01). (^∗^*P* < 0.05 and ^∗∗^*P* < 0.01).

**Figure 2:** Effect of miR-195 expression on CAL-27 cell apoptosis. (a, b) The proportion of apoptotic cells in the miR-195 mimic group is evidently higher than that in the miR-195 control group (*P* < 0.05). (^∗^*P* < 0.05).

**Figure 3:** Correlation between expressions of miR-195 and TLR4 in OSCC cells. (a) Expression of TLR4 in OSCC cells. Compared with HGF, OSCC cells have markedly higher TLR4 mRNA expression (*P* < 0.05). (b) Correlation between expressions of miR-195 and TLR4. Spearman correlation analysis reveals an inverse relation between miR-195 and TLR4 expressions (*P* < 0.001) (^∗^*P* < 0.05).

**Figure 4:** TLR4 is a target of miR-195. (a) Binding sites between miR-195 and TLR4 3′-UTR. (b) Changes in luciferase activity after transfection with mutant-type and wild-type TLR4. The luciferase activity of cells transfected with wild-type TLR4 is significantly lower than that in cells transfected with mutant-type TLR4 (*P* < 0.05). (c) Expression of TLR4 in cells transfected with miR-195. The expression of TLR4 is obviously higher in the miR-195 mimic group than that in the miR-195 control group (*P* < 0.05) (^∗^*P* < 0.05).

**Figure 5:** Effect of miR-195 on NF-*κ*B pathway in OSCC cells. (a) Relative protein expression of p-NF-*κ*B. The p-NF-*κ*B protein expression is remarkably lower in the miR-195 mimic group than that in the miR-195 control group (*P* < 0.05). (b) Changes in p-NF-*κ*B mRNA expression. The p-NF-*κ*B mRNA expression remarkably declines after upregulation of miR-195 (*P* < 0.01) (^∗^*P* < 0.05 and ^∗∗^*P* < 0.01).

## Data Availability

The datasets used and analyzed during the current study are available from the corresponding author on reasonable request.
